The article "MRSA Causing Infections in Hospitals in Greater Metropolitan New York: Major Shift in the Dominant Clonal Type between 1996 and 2014" was published in 2016. Journal: PLoS One.

# MRSA Causing Infections in Hospitals in Greater Metropolitan New York: Major Shift in the Dominant Clonal Type between 1996 and 2014

**DOI:** 10.1371/journal.pone.0156924

**Published:** 2016-06-07

**Authors:** Maria Pardos de la Gandara, Marie Curry, Judith Berger, David Burstein, Phyllis Della-Latta, Virgina Kopetz, John Quale, Eric Spitzer, Rexie Tan, Carl Urban, Guiqing Wang, Susan Whittier, Herminia de Lencastre, Alexander Tomasz

**Affiliations:** 1 Laboratory of Microbiology & Infectious Diseases, The Rockefeller University, New York, New York, United States of America; 2 Division of Infectious Diseases, Saint Barnabas Hospital, Bronx, New York, New York, United States of America; 3 Department of Pathology, Richmond University Medical Center, Staten Island, New York, United States of America; 4 Department of Pathology and Cell Biology, Columbia University Medical Center, New York Presbyterian Hospital, New York, New York, United States of America; 5 Division of Infectious Diseases, SUNY Downstate Medical Center and Kings County Hospital, Brooklyn, New York, United States of America; 6 Department of Pathology, Stony Brook Health Services Center, Stony Brook, New York, United States of America; 7 Department of Microbiology, Saint Barnabas Hospital, Bronx, New York, United States of America; 8 The Dr. James J. Rahal Jr. Division of Infectious Diseases, New York-Presbyterian Queens, Flushing, New York, United States of America; 9 Department of Pathology and Clinical Laboratories, Westchester Medical Center and New York Medical College, Valhalla, New York, United States of America; 10 Clinical Microbiology Service, Columbia University Medical Center, New York Presbyterian Hospital, New York, New York, United States of America; 11 Laboratory of Molecular Genetics, Instituto de Tecnologia Química e Biológica António Xavier (ITQB/UNL), Oeiras, Portugal; Columbia University, UNITED STATES

## Abstract

A surveillance study in 1996 identified the USA100 clone (ST5/SCC*mec*II)–also known as the “New York/Japan” clone—as the most prevalent MRSA causing infections in 12 New York City hospitals. Here we update the epidemiology of MRSA in seven of the same hospitals eighteen years later in 2013/14. Most of the current MRSA isolates (78 of 121) belonged to the MRSA clone USA300 (CC8/SCC*mec*IV) but the USA100 clone–dominant in the 1996 survey–still remained the second most frequent MRSA (25 of the 121 isolates) causing 32% of blood stream infections. The USA300 clone was most common in skin and soft tissue infections (SSTIs) and was associated with 84.5% of SSTIs compared to 5% caused by the USA100 clone. Our data indicate that by 2013/14, the USA300 clone replaced the New York/Japan clone as the most frequent cause of MRSA infections in hospitals in Metropolitan New York. In parallel with this shift in the clonal type of MRSA, there was also a striking change in the types of MRSA infections from 1996 to 2014.

The article "MRSA Causing Infections in Hospitals in Greater Metropolitan New York: Major Shift in the Dominant Clonal Type between 1996 and 2014" was published in 2016. Journal: PLoS One.

## Introduction

*Staphylococcus aureus* has remained a leading cause of infections in hospitals and continues to represent the most frequently identified antibiotic-resistant nosocomial pathogen in many parts of the world [1]. *S*. *aureus* accounted for 12% of all nosocomial infections in the US in 1996, and it still accounts for over 10% of these infections in 2014, in spite of public health controls established in hospitals [2,3]. Moreover, while methicillin-resistant *S*. *aureus* (MRSA) accounted for close to 35% of staphylococcal infections in 1996, this number increased to 60% of all nosocomial *S*. *aureus* infections in more recent years [2–5].

Almost twenty years ago–in 1996 –our laboratory organized a multicenter study to investigate the molecular epidemiology of MRSA in 12 hospitals in Metropolitan New York [2]. At that time, the most prevalent clone, recovered from 113 of 270 MRSA infections (42%), was the ‘New York/Japan’ clone (USA100/ST5/SCC*mec*II), which was also predominant in the neighboring states of Pennsylvania, New Jersey and Connecticut [6]. Subsequently, the same clonal type of MRSA was also identified in hospital infections in Japan [7]. In the United States, this clone has been the predominant MRSA clone in hospitals and healthcare institutions (HA-MRSA) countrywide over the last fifteen years [8,9].

According to the National Nosocomial Infections Surveillance, the rates of MRSA infection in hospitals in New York City have been increasing from 619 cases in 1997 (35% of all *S*. *aureus* infections in hospitals) to 3,470 cases in 2004 (60% of all *S*. *aureus* infections in hospitals) [10]. In parallel, the frequency of MRSA infections in hospitals due to community-associated MRSA (CA-MRSA) clones has also increased from 18% in 1997 to 25% in 2004 [9,11].

On the other hand, the New York State Department of Health reported a decrease in the number of hospital MRSA infections during the past seven years: MRSA infections in colon surgery decreased from 84 cases in 2008 to 74 in 2013; coronary bypass infections decreased from 55 in 2008 to 24 in 2013; and central-catheter-associated bloodstream infections in children and adults decreased from 73 in 2008 to 20 in 2013. However, the number of central-catheter-associated bloodstream infections in neonatal intensive care units due to MRSA increased from three in 2008 to ten in 2013 [12,13].

The latest report from the Active Bacterial Core Surveillance Program (ABCSP) described a reduction in the national incidence of hospital acquired MRSA invasive infections between 2005 and 2011. However, the authors described an increased risk of recurrence among healthcare-associated community-onset infections and a very limited change in the rate of community-associated infections [14].

The article "MRSA Causing Infections in Hospitals in Greater Metropolitan New York: Major Shift in the Dominant Clonal Type between 1996 and 2014" was published in 2016. Journal: PLoS One.

In the present study we report on the clonal types of MRSA isolates recovered from infections in several of the same hospitals in New York City that participated in the 1996/98 surveillance.

## Materials and Methods

The study was reviewed and approved by the Institutional Review Board (IRB) at The Rockefeller University.

### Hospital network

The eight hospitals that participated in this study and their location within the greater New York City area are shown in **Fig 1**. These hospitals were as follows: VA Hospital (IV) and Kings County Hospital (XIII) in Brooklyn; Columbia University Medical Center (II) in Manhattan; New York-Presbyterian Queens (VI) in Queens; St. Barnabas Hospital (IX) in the Bronx; Richmond University Medical Center (X) in Staten Island; Stony Brook Health Sciences Center (XI) in Long Island; and Westchester Medical Center (XII) in Valhalla. Seven of these eight hospitals (all except Kings County Hospital) also participated in the previous surveillance study in 1996.

**Fig 1:** Geographic location of hospitals that participated in the two surveillance studies. Numbers from I to XII represent the 12 hospitals that collaborated with the Rockefeller University in the 1996 surveillance study and circled in gray are the 8 hospitals that collaborated again in 2013/14. Hospital XIII was added to the participating hospitals in 2013/14.

### Source of MRSA isolates

MRSA isolates were obtained from the Pathology Departments of the participating hospitals. Individual centers were asked to submit single patient MRSA isolates obtained from inpatient cultures during an extended period from January 2013 to August 2014. The number of specimens provided by each institution was a convenience figure, calculated to be proportional to the sample size of 1996, the rates of sterile site infections in 2013 and the number of inpatient beds in each hospital (**Table 1**). The 121 bacterial isolates were inoculated on BHI, chocolate slants or blood agar plates for room temperature transportation to the Laboratory of Microbiology and Infectious Diseases at The Rockefeller University on the same day, following the U.S. Department of Transportation Pipeline and Hazardous Materials Safety Administration guidelines [15]. All isolates were grown overnight on Mannitol Salt Agar plates (MSA, Difco, BBL, Becton Dickinson, Franklin Lakes, NJ, USA) and were tested for coagulase agglutination (Staphaurex, Thermo Fisher Scientific, Lenexa, KS, USA) to confirm species identification.

The article "MRSA Causing Infections in Hospitals in Greater Metropolitan New York: Major Shift in the Dominant Clonal Type between 1996 and 2014" was published in 2016. Journal: PLoS One.

**Table 1:** MRSA specimens provided by the participating hospitals.

			1996		2013/14	
Hospital	Location (Fig 1)	Neighborhood	# MRSA isolates analyzed	Beds	# MRSA isolates analyzed	Beds
Columbia University Medical Center	II	Manhattan	20	1475	39	1200
Kings County Hospital	XIII	Brooklyn	—	—	9	700
VA Hospital	IV	Brooklyn	15	324	2	340
New York-Presbyterian Queens Center	VI	Queens	28	487	9	539
St. Barnabas Hospital	IX	Bronx	18	458	8	417
Richmond University Medical Center	X	Staten Island	27	638	35	450
Stony Brook Health Sciences Center	XI	Stony Brook	19	536	10	597
Westchester Medical Center	XII	Valhalla	17	639	9	635
Total			144	4557	121	4878

Location: Roman numbering identifies the particular hospitals in Fig 1 and also corresponds to the listing in the 1996 surveillance. Some hospitals that collaborated at that time did not participate in 2013/14, due to closure or association with other institutions.

# MRSA isolates analyzed: isolates of methicillin-resistant *S*. *aureus* provided by each hospital.

# Beds: number of inpatient beds per hospital.

### Antimicrobial susceptibility testing

MRSA antibiograms were performed by either micro-dilution, E-test or disk-diffusion methods, following the Clinical and Laboratory Standards Institute (CLSI) recommendations [16]. All specimens were tested for susceptibility to a number of antibiotics at the particular hospital providing the strains. Since not all hospitals tested the same antibiotics, in order to allow comparisons, additional tests were performed at the Rockefeller University so all specimens were tested at least with the following antibiotics: penicillin, oxacillin, ciprofloxacin, clindamycin, erythromycin, gentamicin, rifampicin, tetracycline, trimethoprim/sulfamethoxazole, linezolid, nitrofurantoin, chloramphenicol, daptomycin, vancomycin and mupirocin.

### Molecular identification: *spa* typing, MLST, PFGE, SCC*mec* typing

Molecular characterization of the 121 MRSA isolates was performed initially by *spa* typing as described [17] and using the RIDOM web server (http://spaserver.ridom.de/) for assignment of *spa* types. The *spa* server was also used to predict sequence types (ST). MLST was performed as previously described [18] when the *spa* server and the bibliography did not provide STs to the *spa* types obtained. Assignment of STs was done by DNA amplification and sequencing of seven housekeeping genes (*arcC*, *aroE*, *glpF*, *gmk*, *pta*, *tpi*, *yqiL*) using the online MLST database (http://www.mlst.net/). Clonal Complexes were determined for the STs [19].

The article "MRSA Causing Infections in Hospitals in Greater Metropolitan New York: Major Shift in the Dominant Clonal Type between 1996 and 2014" was published in 2016. Journal: PLoS One.

PFGE was performed to further confirm the relatedness of MRSA isolates belonging to the same clonal complex. Bacterial DNA was restricted with *Sma*I enzyme and the resulting fragments were separated by electrophoresis [20]. Band patterns were compared manually following guidelines to confirm classification [21,22].

The classification of staphylococcal cassette chromosome *mec* (SCC*mec*) carried by the isolates was determined using multiplex PCR, following previous guidelines [23,24]. Ambiguous results were further tested by amplification of the *ccrB* gene [25] and comparing the sequences obtained with the online database available at the Laboratory of Molecular Genetics at Instituto de Tecnologia Quimica e Biologica (ITQB) in Portugal. SCC*mec* was considered non-typable (NT) when it was not possible to ascertain a class of *mec* complex and/or a type of *ccrB*. SCC*mec* type IV subtyping was also performed by multiplex PCR as previously described [26].

### Molecular characterization: detection of *mecA*, PVL, and ACME

The *mecA* gene, responsible for resistance to oxacillin and other beta-lactam antibiotics and the *lukS* and *lukF* genes (which encode PVL, the Panton-Valentine leukocidin) were identified by PCR [27,28].

The arginine catabolic mobile element (ACME) element was identified and typed using primers that target its two main loci (*arcA* and *opp3*) in USA300 strain FPR3757 [29] and classified according to its structure: type I (*arc* and *opp3* operons), type II (*arc* operon only) and type III (*opp3* operon only)[30].

## Results

Of the 12 New York City area hospitals that participated in the original surveillance study in 1996, seven also took part in the study described here. The list of participating hospitals is in **Table 1** and their location is shown in **Fig 1**. Four of the hospitals that were part of the original study no longer exist: they closed or merged with other institutions. The molecular epidemiology of MRSA in the New York Presbyterian Hospital/Cornell Medical Center will be described in a separate communication.

The total number of beds in the participating hospitals was 4,878, ranging from 1,200 beds in hospital II to 340 in hospital IV. A total of 121 MRSA isolates were obtained in the surveillance study. With a median of ten samples per hospital, each center provided MRSA isolates ranging in number from eight to 39 (**Table 1**). Most MRSA (26%) was recovered from Medical services (Internal Medicine, Neurology, Cardiology, Oncology and Nephrology) and the second most frequent source was Pediatrics (25%). Information regarding the service attended at the time of the sample collection was not available for 12 of the samples: three samples originating from the VA Hospital in Brooklyn and nine samples from the New York-Presbyterian Queens Hospital in Flushing. The age of patients ranged from 0 (sample taken at the time of delivery) to 94 years with a median age of 54 years old; 32% of patients were >60 years old but the age-group most often involved with MRSA infections was the 0–9 years group (21 cases). For a single patient the age was not available. Isolates were recovered from a variety of sources: 58 SSTIs (skin and soft tissue infections), 50 blood cultures, four respiratory samples, two samples from a placental infection (mother and child), one urine sample, one cerebrospinal fluid sample, and one synovial fluid extraction. No biological source was available for three samples from the VA Hospital in Brooklyn and for one sample from the Richmond University Medical Center in Staten Island at the time of the molecular analysis.

The article "MRSA Causing Infections in Hospitals in Greater Metropolitan New York: Major Shift in the Dominant Clonal Type between 1996 and 2014" was published in 2016. Journal: PLoS One.

Of the 121 isolates characterized 86 (71%) presented a multi-drug resistant (MDR) phenotype, i.e, they were resistant to at least three different classes of antibiotics. These MDR isolates included 20 of the 25 (80%) USA100 strains and 54 of the 78 (69%) USA300 strains. One isolate belonging to the USA100 clone was resistant to seven different antibiotics. Isolates belonging to clone USA100 were more frequently than USA300 isolates resistant to quinolones (92% vs 72%), clindamycin (84% vs 17%), gentamicin (8% vs 0%), rifampicin (8% vs 1%), daptomycin (12% vs 5%), and trimethoprim/sulfamethoxazole (12% vs 4%), while isolates of the USA300 clone were more often resistant to tetracycline (3% vs 0%) and to mupirocin (13% vs 8%). Both clones showed similar proportion of isolates resistant to erythromycin (92% of USA100 vs 90% of USA300 isolates). No isolates resistant to linezolid, nitrofurantoin, chloramphenicol or vancomycin were detected. Ten of the 13 isolates showing high resistance against mupirocin (MIC ≥ 1024 μg/ml) belonged to the USA300 clone. The antibiotic resistance patterns of MRSA isolates are shown in **Table 2**.

**Table 2:** Antimicrobial resistance profiles of strains characterized in the study.

	TOTAL			USA100			USA300			Others		
	n	No. R	% R	n	No. R	% R	n	No. R	% R	n	No. R	% R
OXA	121	121	100%	25	25	100%	78	78	100%	18	18	100%
CIP	121	90	**74%**	25	23	**92%**	78	56	**72%**	18	11	**61%**
CLI	121	37	**31%**	25	21	**84%**	78	13	**17%**	18	3	**17%**
ERY	121	104	**86%**	25	23	**92%**	78	70	**90%**	18	11	**61%**
GEN	121	3	**2%**	25	2	**8%**	78	0	**0%**	18	1	**6%**
RIF	121	4	**3%**	25	2	**8%**	78	1	**1%**	18	1	**6%**
TET	121	5	**4%**	25	0	**0%**	78	2	**3%**	18	3	**17%**
SXT	121	11	**9%**	25	3	**12%**	78	3	**4%**	18	5	**28%**
MUP	121	13	**11%**	25	2	**8%**	78	10	**13%**	18	1	**6%**
DAP	121	7	**6%**	25	3	**12%**	78	4	**5%**	18	0	**0%**
LZD	121	0	0%	25	0	0%	78	0	0%	18	0	0%
NIT	121	0	0%	25	0	0%	78	0	0%	18	0	0%
VAN	121	0	0%	25	0	0%	78	0	0%	18	0	0%
CHL	121	0	0%	25	0	0%	78	0	0%	18	0	0%

OXA: oxacillin; CIP: ciprofloxacin; CLI: clindamycin; ERY: erythromycin; GEN: gentamicin; RIF: rifampin; TET: tetracycline; SXT: trimethoprim/sulfamethoxazole; MUP: mupirocin; DAP: daptomycin; LZD: linezolid; NIT: nitrofurantoin; VAN: vancomycin; CHL: chloramphenicol.

The article "MRSA Causing Infections in Hospitals in Greater Metropolitan New York: Major Shift in the Dominant Clonal Type between 1996 and 2014" was published in 2016. Journal: PLoS One.

**No. R**: number of isolates resistant to a specific antibiotic; **n**: number of strains analyzed; **%R**: percentage of resistant isolates in each group. Highlighted are those antibiotics to which either USA100 or USA300 are more prone to be resistant.

The majority of the MRSA isolates (86 of the total of 121) belonged to a variety of community-associated MRSA clones, most of these (78 isolates) belonged to the USA300 clone (ST8/SCC*mec*IV/PVL^±^/ACME^±^). Three were representatives of USA700 (ST72/SCC*mec*IV/ PVL^-^/ACME^—^); two were USA1100 (ST30/SCC*mec*IV/PVL^+^/ACME^—^); one was USA400 (ST1/SCC*mec*IV/PVL^+^/ACME^—^); one was USA1000 (ST59/SCC*mec*IV/PVL^—^/ACME^—^); and one isolate was ST88/SCC*mec*IVa/PVL^+^/ACME^—^.

Molecular characterization of MRSA identified twenty-eight different *spa* types, which could be assigned to seven ST types. Of the total of 121 MRSA characterized, 35 belonged to typical hospital-associated clones: twenty-three of these were representatives of the USA100 (‘New York/Japan’) clone (ST5/SCC*mec*II/PVL^—^/ACME^—^) and two additional isolates shared the same PFGE/MLST/PVL/ACME profile but had a non-typable SCC*mec* cassette. There were three isolates belonging to the USA800 (‘Pediatric’) clone (ST5/SCC*mec*IV/PVL^—^/ACME^—^); six isolates belonged to the USA500 clone (ST8/SCC*mec*IV/PVL^—^/ACME^—^) and one isolate had the same PFGE/MLST/PVL/ACME profile as USA500 but carried a non-typable SCC*mec* cassette.

All but six isolates (72 of 78) belonging to the USA300 clone had the ACME virulence determinant but no strains belonging to the other clones carried ACME. The great majority (74 of 78) of USA300 isolates encoded the PVL toxin; only four isolates belonging to clones other than USA300 carried these genetic determinants. These were two isolates of the USA1100, one ST88 isolate and one USA400 isolate. None of the 35 HA-MRSA isolates carried either ACME or PVL determinants.

The currently major USA300 clone was represented by several *spa* variants (11 *spa* types) with t008 as the most prevalent type (63 of 78 isolates, 80.77%).

The previously dominant MRSA clone USA100 (‘New York/Japan’ clone) was represented by 25 isolates, 20 of which (80%) had the t002 *spa* type. The *spa* types of the remaining clones are shown in Table 3.

The article "MRSA Causing Infections in Hospitals in Greater Metropolitan New York: Major Shift in the Dominant Clonal Type between 1996 and 2014" was published in 2016. Journal: PLoS One.

**Table 3:** Distribution of MRSA clones and the different *spa* types and SCCmec types identified in this study.

MRSA Clones	n^a^	associated *spa* types ^b^	SCC*mec* types
USA100 (NY/Japan)	25	t002 (20), t062 (1), t071 (1), t088 (1), t306 (1), t856 (1)	II, NT^d^ (t002)
USA300	78	t008 (62), t024 (1), t051 (1), t068 (2), t121 (3), t211 (3), t351 (1), t723 (1), t1635 (1), t2229 (1), t3908 (2)	IVa
USA400	1	t128 (1)	IVa
USA500	7	t008 (1), t064 (2), t211 (1), t394 (1), t1774 (1), t13975 (1)^c^	IVg, NT (t211)
USA700	3	t126 (1), t901 (1), t1346 (1)	IVa (t126), IVh (t901), NT (t1346)
USA800	3	t002 (3)	IVh, IVnst^e^
USA1000	1	t216 (1)	IVa
USA1100	2	t665 (2)	IVa
ST88	1	t692 (1)	IVa
Total:	121		

^a^ Number of MRSA isolates belonging to a particular clone

^b^ Numbers in parenthesis represent the number of isolates with a particular *spa* type

^c^ t13975 was a new *spa* type identified for the first time in this study

^d^ Non-typable

^e^ Non-sub-typable

The staphylococcal cassette chromosome (SCC*mec*) was also characterized: all isolates carried variants of the type IV cassette, except the USA100 (‘New York/Japan’) isolates, which carried the SCC*mec*-II characteristic of this clone; the cassette was non-typable for two isolates belonging to the USA100 clone (t002) and one USA500 isolate (t211) (**Table 3).**

## Discussion

The total number of beds in the hospitals collaborating in the 1996 surveillance study was 5,117 as compared to the 4,878 beds in the hospitals participating in the current (2013/14) surveillance. The total number of MRSA isolates characterized in 1996 was 270 and 121 in 2013/14. In the study described here, the patients were younger than in the previous surveillance: while 58% of patients were >60 years old in the 1996 study, that age group represented only 32% in the current in 2013/14 study. Medical services are still frequently affected by MRSA infections. In 1996 this group had 71% of all isolates although in the current surveillance this number was reduced to 26%. The second most frequently affected service—Pediatrics—had 25% of the MRSA cases in the present study.

Comparison of the results of the surveillance study described here to the surveillance conducted 15 years earlier, in 1996 [2] show several striking differences. In 1996 a single clone, USA100 (‘New York/Japan’) was responsible for 42% of all MRSA infections in 12 New York City hospitals [2]. In the study described here, with MRSA isolates collected in 2013/14, a different clone—USA300—was involved with most (64.4%) MRSA infections (**Table 4**). The other strains collected in 2013/2014 belonged to three different HA-MRSA clones: 25 were representatives of the USA100 clone, seven isolates of USA500 and three to the USA800 clone. The remaining 86 isolates belonged to six community-acquired MRSA lineages: USA300 (78 isolates), USA700 (three isolates), USA1100 (two isolates), USA400 (one isolate), USA1000 (one isolate) and one ST88 isolate.

The article "MRSA Causing Infections in Hospitals in Greater Metropolitan New York: Major Shift in the Dominant Clonal Type between 1996 and 2014" was published in 2016. Journal: PLoS One.

**Table 4:** Representation of MRSA clones USA100, USA300 and other clonal types in New York City area hospitals during the two surveillance periods.

		USA100 (‘NY/Japan clone) ST5, SCC*mec*II				USA300 clone ST8, SCC*mec*IVa		Other Clonal Types		Total No of MRSA isolates*
		1996		2013/14						
Hospital	Location**	No	%^#^	No	%^#^	No	%^#^	No(ǂ)	%^#^	No
Columbia Presbyterian Medical Ctr	II	5	25	1	2.5	34	87.0	4 (3)	10.2	**39**
Kings County Hospital	XIII	—	—	3	37.5	2	80.0	3 (2)	37.5	**8**
VA Hospital	IV	9	60	1	33.3	2	66.6	0	—	**3**
New York-Presbyterian Queens	VI	15	53.6	1	11.1	5	55.5	3 (3)	33.3	**9**
St. Barnabas Hospital	IX	5	27.8	2	25.0	5	62.5	1	12.5	**8**
Richmond University Medical Ctr	X	9	33.3	11	31.4	20	57.1	4 (3)	11.4	**35**
Stony Brook Health Sciences Center	XI	14	73.7	5	50.0	3	30.0	2 (2)	20.0	**10**
Westchester Medical Center	XII	8	47.1	1	10.0	7	80.0	1	10.0	**9**
**TOTAL**		**113**	**41.9**	**25**	**20.5**	**78**	**64.7**	**18**	**14.7**	**121**

*Total number of MRSA isolates recovered and tested in 2013/14 surveillance

**See Fig 1

^**#**^ Clonal type in percentage of all MRSA identified in the hospitals

**(ǂ)** Numbers in parentheses indicate the number of different clonal types of MRSA identified in the particular hospital.

The change in clonal type of MRSA was also accompanied by a change in the type of infections. While in 1996 MRSA was mainly recovered from the respiratory tract (44%), most of the MRSA infections in 2013/14 were skin and soft tissues (SSTIs) (48%). Also, bacteremia/sepsis has increased from 17.5% of MRSA infections in 1996 to 41.3% in 2013/14. **Fig 2** illustrates the change in the types of lesions and **Fig 3** shows the predominant MRSA clones in 1996 and in 2013/14.

**Fig 2:** Change in the clinical sources of MRSA from 1996 to 2014. ‘Respiratory tract’: lower respiratory tract (including sputum and bronch-alveolar lavage) and sinusitis and pleural fluid. ‘Other’: any other biological specimen from which MRSA was isolated at any of the hospitals including the urinary tract, cerebro-spinal fluid, synovial fluid, placental biopsy and unlisted specimens.

**Fig 3:** **PFGE profiles of hospital isolates representing the major clonal types of MRSA identified in the 1996 (A) and the 2013/14 study (B). (A)** PFGE of USA100 isolates in 1996 [2]**. (B)** PFGE of USA300 isolates in 2013/14. Migration on TBE-agarose gel after digestion with *SmaI* restriction enzyme. USA100 (‘New York/Japan’) was the predominant clone in 1996, and the second most frequent clone in 2013–14. The roman numbers on each strain indicate the hospital in which they were isolated.

The article "MRSA Causing Infections in Hospitals in Greater Metropolitan New York: Major Shift in the Dominant Clonal Type between 1996 and 2014" was published in 2016. Journal: PLoS One.

While the MRSA clone USA300 is known to have a strong association with SSTIs [31,32], there is no specific association known between the USA100 clone and respiratory infections. A recent report from the CDC (Emerging Infections Program Healthcare-Associated Infections and Antimicrobial Use Prevalence Survey Team) concluded that *S*. *aureus* (together with *Klebsiella oxytoca* and *K*. *pneumoniae*) were currently the main pathogens responsible for respiratory tract and skin and soft infections [33].

As to the possible mechanism that has led to the changed clonal types between the current and the previous (1996) surveillance, we hypothesize that the infection control mechanisms introduced in the healthcare system may have succeeded in controlling the spread of HA-MRSA clones like USA100, while the entry and spread of community-associated MRSA strains in hospitals may be responsible for the increase of SSTIs and secondary bacteremia/sepsis [9,34]. Recent reports indicate that the number of invasive MRSA infections decreased in the United States in 2011 as compared to 2005, but more MRSA infections occurred in the community than during hospitalization in 2011 [35,36]. The hospital as a source of MRSA infections seems to have become better controlled, but the frequency of MRSA infections in the community appears to be increasing. Several other studies have documented the “escape” of MRSA clones from hospitals to the healthy community and to public transportation [37,38].

New clones circulating in both the community and hospitals also come with a change in patient demographics, i.e., younger patients presenting with different types of infections and with an increase in SSTIs and blood infections and decrease in respiratory infections caused by MRSA [3,39,40].

The change in clonal type of MRSA strains in hospitals between the two studies in 1996 and 2013/14 is also associated with a change in the pattern of antibiotic resistance. In the study performed in 1996, where the USA100 clone was predominant, up to 96% of strains analyzed were resistant to ciprofloxacin. In 2013/14 only 74% of strains showed this resistance phenotype. This may be due to the current predominance of strains belonging to the USA300 clone (72% of them resistant to ciprofloxacin), as resistance to quinolones reached 92% of strains belonging to the USA100 clone. Similarly, resistance to clindamycin affected 88% of strains in 1996, while only 31% of strains in 2013/14 were resistant to this antibiotic, and 84% of the clindamycin resistant strains belonged to the USA100 clone. In addition, in 1996 it was reported that 58% of the characterized strains were resistant to gentamicin while in 2013/14 only three isolates showed this phenotype.

The article "MRSA Causing Infections in Hospitals in Greater Metropolitan New York: Major Shift in the Dominant Clonal Type between 1996 and 2014" was published in 2016. Journal: PLoS One.

Following the recommendations of the Infectious Diseases Society of America [41] vancomycin has been the antibiotic of choice against MRSA invasive infections in hospitalized patients in each of the hospitals participating in this study. All MRSA isolates characterized in this study were susceptible to this antibiotic. Other therapeutic options such as daptomycin, clindamycin, rifampin, gentamicin or trimethoprim/sulfamethoxazole have also been used–alone or in combination–and the high rates of resistance observed in our study to these antibiotics underlines the importance of keeping track of the drug resistance mechanisms of MRSA strains circulating in a hospital–in order to prevent possible treatment failures. It should also be noted that a number of isolates belonging to the currently predominant MRSA clone USA300 –also show resistance to mupirocin (see **Table 2**)–an agent frequently used for decolonization and topical treatment [42].

It is interesting that the SCC*mec* type IV, common in community-associated MRSA (CA-MRSA), is also present in some HA-MRSA clones like USA500 or USA800. As many as 98 out of the 121 hospital isolates studied here were harboring the type IV SCC*mec* cassette, compared to the 23 isolates belonging to USA100 which carried the SCC*mec* cassette type II. The smaller size of the type IV cassette has been postulated as an evolutionary advantage for MRSA clones carrying this cassette [8,9,31].

The virulence factors ACME and PVL are often carried by CA-MRSA strains even when these clones are recovered in the hospital setting. In our study, ACME was exclusively carried by USA300 strains while the PVL was present in other CA-MRSA clones as well.

Several factors may have contributed to the shift in the clonal type of MRSA from the “New York/Japan clone” dominant in the 1996 surveillance to the MRSA clone USA300 most prevalent in 2013/14. These factors may include the smaller (type IV) SCC*mec* cassette carried by the USA300 clone and also the presence of virulence factors like ACME and PVL in the MRSA clone USA300, which seems to have emerged as the most prevalent clone both in hospitals and in the community [11,31,43].
